RETRACTED

# Naringin protects endothelial cells from apoptosis and inflammation by regulating the Hippo-YAP Pathway

**DOI:** 10.1042/BSR20193431

**Published:** 2020-03-04

**Authors:** Hui Zhao, Meirong Liu, Hui Liu, Rong Suo, Chengzhi Lu

**Affiliations:** 1 Department of Cardiology, First Center Clinic College of Tianjin Medical University, Tianjin 300192, China; 2 Department of Respiration, Tianjin Hospita, Tianjin 300211, China; 3 Department of Cardiology, Tianjin Hospital, Tianjin 300211, China

**Keywords:** apoptosis, Endothelial cells, Hippo-YAP Pathway, inflammation, Naringin

## Abstract

Atherosclerosis is the primary cause of several cardiovascular diseases. Oxidized low-density lipoprotein (ox-LDL)-induced apoptosis, endothelial–mesenchymal transition (EndMT), and inflammation are crucial for the progression of cardiovascular diseases, including atherosclerosis. Naringin, a major compound from tomatoes, grapefruits, and related citrus, reportedly exhibits potential protective effects during atherosclerosis development; however, its effect on ox-LDL-induced human umbilical vein endothelial cell (HUVEC) damage remains unknown. In the present study, we investigated the anti-apoptotic and anti-inflammatory activities of naringin against ox-LDL-induced endothelial cells, and the underlying mechanism. Naringin pretreatment significantly and concentration-dependently inhibited ox-LDL-induced cell injury and apoptosis. Additionally, naringin restored endothelial barrier integrity by preventing VE-cadherin disassembly and F-actin remodeling, and down-regulated pro-inflammatory factors like IL-1β, IL-6, and IL-18, in the HUVECs. We also demonstrated that naringin treatment restored ox-LDL-induced YAP (yes-associated protein) down-regulation, given the YAP-shRNA attenuated cytoprotective effect of naringin on ox-LDL-induced endothelial cell injury and apoptosis. Collectively, our data indicate that naringin reversed ox-LDL-triggered HUVEC apoptosis, EndMT, and inflammation by inhibiting the YAP pathway. Therefore, naringin may have a therapeutic effect on endothelial injury-related disorders.

## Introduction

Atherosclerosis is the predominant cause of cardiovascular diseases, and is becoming a global concern, owing to its high prevalence [1]. Endothelial injury and apoptosis are the main pathological processes of atherosclerosis, known to trigger thrombosis and accelerate atherosclerotic plaque formation [2]. The arterial deposition of ox-LDL cholesterol is closely associated with atherosclerosis-related morbidity [3].

Accumulating evidence indicate the common occurrence of endothelial–mesenchymal transition (EndMT) in atherosclerosis [4]. EndMT is characterized by specific endothelial marker loss, and mesenchymal marker acquisition [5]. The loss of morphological and functional vascular endothelial cell integrity is closely related to cell inflammation and apoptosis in atherosclerosis [6,7]. Ox-LDL promotes the formation and development of atherosclerotic plaques, by inducing vascular endothelial inflammation and apoptosis [8]. Therapeutic strategies against vascular endothelial cell EndMT, inflammation, and apoptosis may lead to the remission of endothelial-related pathology [9].

RETRACTED

Naringin is a major compound extracted from tomatoes, grapefruits, and related citrus fruits [10]. It exhibits potential protective effects against atherosclerosis development [11,12]. Pharmacological investigations have shown that naringin has anti-inflammatory, anti-oxidant, anti-apoptotic, and hepato-protective effects [13,14]. However, no reports exist on its anti-apoptotic and anti-inflammatory effects in ox-LDL-induced injury, in human umbilical vein endothelial cells (HUVECs).

The yes-associated protein 1 (YAP) is the most critical downstream effector in the Hippo signaling cascade, and is essential for physiological and pathological processes [15]. The Hippo–YAP pathway is a kinase cascade consisting of a series of protein kinases and transcription factors [16]. YAP is important for cell proliferation, endothelial cell activation, and vascular inflammation [17].

Thus, in the present study, we established an *in vitro* atherosclerosis model, by exposing endothelial cells to ox-LDL. The effects of naringin on ox-LDL-induced endothelial injury, apoptosis, and inflammation were investigated. We also quantitatively analyzed the mRNA expressions of YAP and inflammatory cytokines, such as IL-1β, IL-6, and IL-18. It is our hope that the present study will improve the value of naringin as a potential candidate for ox-LDL-induced endothelial injury treatment in atherosclerosis and other cardiovascular diseases.

## Materials and methods

### Cell culture and treatment

HUVECs were purchased from ScienCell (San Diego, CA, U.S.A.), and maintained in ECM (San Diego, CA, U.S.A.) containing 10% heat-inactivated fetal bovine serum (Gibco, Carlsbad, CA), 1% penicillin/streptomycin solution, and 1% endothelial cell growth supplement, at 37°C in 5% CO_2_. To evaluate the cell protective effect of naringin on ox-LDL (Yiyuan Biotechnologies, Guangzhou, China)-induced HUVECs, cells were randomly divided into three groups: the naringin-treated group where cells were exposed to naringin at 10, 50, 100 and 200 μM for 24 h; the ox-LDL-treated group where cells were exposed to ox-LDL at 20, 40, 60 and 80 μg/ml for 24 h; and the ox-LDL+ naringin-treated group where cells were pretreated with naringin for 2 h, and then incubated with ox-LDL for 24 h. Each group had a minimum of three replicated wells. Subsequently, cells were harvested and extracted for further analyses.

RETRACTED

### Cell viability assay

The cell counting Kit-8 CCK-8 (Dojindo, Kumamoto, Japan) was used to test the cell viability, following the manufacturer’s instructions. Cells were plated onto 96-well plates (4 × 10^4^ cells/well), each well was supplemented with 10 μl of CCK-8 solutions for 2 h at 37°C, and the cell absorbencies measured at 450 nm, using a spectrophotometer.

### Lactate dehydrogenase (LDH) release assay

To evaluate cell injury, cytosolic LDH released into culture medium was measured, as previously described [18]. After the 2 h naringin pretreatment, followed by 24 h incubation with 80 μg/ml ox-LDL, medium was collected from each well. Supernatants were obtained by centrifugation at 12,000 × ***g*** at 4°C for 10 min. LDH release was determined using an LDH assay kit (Jiancheng Bioengineering Institute, Nanjing, China), following the manufacturer’s instructions. LDH activity was determined via a colorimetric assay using an absorbance wavelength of 492 nm in a spectrophotometer (Bio-Rad Laboratories).

### TUNEL staining

The TUNEL apoptosis determination kit (Beyotime, Jiangsu, China) was used to detect apoptotic cells in HUVECs, following the manufacturer’s instructions. Briefly, after all treatments, cells were washed with PBS, fixed with 1% buffered formaldehyde, followed by fixation in an ethanol and acetic acid mixture. The fixed cells were stained using fluorescein-conjugated TUNEL, and the cell nuclei were stained with DAPI. The TUNEL-positive cells were observed under a fluorescence microscope (Leica DM4000, Germany). The apoptotic rate was quantified by counting TUNEL positive cells from six random fields, and the values were expressed as a percentage of the total number of cells.

### Annexin-V/PI staining and flow cytometry

Apoptosis was measured by flow cytometry. HUVECs (5 × 10^5^ cells) were collected by centrifugation at 1000 × ***g*** at 4°C, for 10 min, followed by two rounds of cell pellet washing with HEPES-buffered saline. The cells were then fixed with 70% ice-cold methanol at 4°C for 30 min. After re-suspending with the binding buffer, cells were stained with 10 μl Annexin V-fluorescein isothiocyanate (FITC), and 5 μl propidium iodide (PI) for 10 min, in the dark. The stained cells were analyzed by flow cytometry (FACSCalibur; BD Biosciences, U.S.A.). The measurements were recorded at least three times in individual experiments.

### Quantitative real-time PCR

TRIzol reagent (Invitrogen, Carlsbad, CA, U.S.A.) was used to extract total RNA. The primer sequences were designed based on GenBank cDNA sequences. A cDNA Synthesis Kit (Applied Biosystems, Foster City, CA, U.S.A.) was used to reverse transcribe 1 µg of total RNA into cDNA. Levels of IL-1β, IL-6, IL-18, YAP, and GAPDH (internal control) mRNAs were analyzed using the SYBR RT-PCR Kit (Takara, Dalian, China). Forty PCR cycles were conducted at 95°C for 30 s and 60°C for 30 s, preceded by 1 min at 95°C for polymerase activation. Quantitative PCR (qPCR) was performed using the MiniOpticon qPCR detection system (Bio-Rad Laboratories). The 2^−ΔΔCT^ method was adopted to calculate the relative quantification. Primer sequences are shown in Table 1.

RETRACTED

**Table 1:** Primers used in the present study

Gene		Primer sequence(5′-3′)
GAPDH	Forward	CACATGGCCTCCAAGGAGTA
	Reverse	TCCCCTCTTCAAGGGGTCTA
IL-1β	Forward	TTCCTGTTGTCTACACCAATGC
	Reverse	CGGGCTTTAAGTGAGTAGGAGA
IL-6	Forward	TCTCTCCGCAAGAGACTTCCA
	Reverse	ATACTGGTCTGTTGTGGGTGG
IL-18	Forward	TTCCTCTTCCCGAAGCTGTGTAGACTGC
	Reverse	CCGCTTTAGCAGCCAGAGTTGGCAGCCAGG
YAP	Forward	GTTGGGAGATGGCAAAGACA
	Reverse	ACGTTCATCTGGGACAGCAT

### Transfection

HUVECs (4 × 10^5^ cells/well) were seeded onto a 6-well plate and transfected with YAP shRNA (5′-CCCAGTTAAATGTTCACCAAT-3′), and control shRNA (OriGene Technologies Inc, U.S.A.), using Lipofectamine 2000 (Invitrogen, Carlsbad, CA, U.S.A.), following the manufacturer’s instructions. After 6 h, the transfection mixture was replaced with fresh growth medium. Subsequent experiments with transfected cells were performed after 48 h transfection.

### Western blotting

HUVECs were collected and lysed in RadioImmunoprecipitation Assay (RIPA) buffer (Thermo Fisher Scientific, Waltham, MA, U.S.A.), with PMSF lysis buffer. The protein concentration was quantified using the bicinchoninic acid protein assay kit (Beyotime Biotechnology, Shanghai, China). Equal protein amounts (30 μg) were separated by loading on a 12% gel for SDS-PAGE, and transferring the separated protein onto PVDF membranes (EMD Millipore, Billerica, MA, U.S.A.). Blots were blocked and immunoblotted with VE-Cadherin (Cell Signal, USA, 1:1000, ab7652), F-actin (Cell Signal, U.S.A., 1:500, ab2357), YAP (Abcam, U.S.A., 1:1000, ab48635), and GAPDH (Abcam, U.S.A., 1:1000, ab4563). The membranes were then incubated with the corresponding secondary horseradish peroxidase–conjugated secondary antibodies (Abcam, U.S.A.) for 2 h at 25°C. The protein bands were visualized using ECL chemiluminescence, and quantified by Image-Pro Plus 6.0 (Media Cybernetics, Bethesda, MD, U.S.A.). Separation of F-actin from G-actin pool in HUVECs were determined using the G-actin/F-actin in vivo assay kit (Cytoskeleton, Inc., Denver, CO), according to the manufacturer’s instructions. Briefly, HUVECs were lysed in F-actin stabilization buffer, following high-speed centrifugation (100,000 × ***g*** spin for 1 h at 37°C), the pellet (F-actin) was resuspended with a depolymerizing agent and then mixed with SDS loading buffer, electro-transferred to PVDF and probed with anti-F-actin antibody.

RETRACTED

### Immunofluorescent staining

HUVECs were cultured on glass slides, washed in PBS, and fixed with 4% paraformaldehyde for 30 min. The cells were then permeabilized with PBS containing 0.5% Triton X-100 for 15 min. The VE-Cadherin (Cell Signal, U.S.A., 1:1000, ab7652) or F-actin (Cell Signal, U.S.A., 1:500, ab2357) antibody was applied to the coverslip and incubated overnight at 4°C. After three rounds of PBS washes, the fluorescent secondary antibody (Beyotime, China, 1:500, ab5468) was added and incubated for 1 h at 25°C. Following three additional PBS washes, cell nuclei were co-stained with DAPI. Images were captured using a fluorescence microscope (Nikon, Tokyo, Japan).

### Statistical analyses

Data are presented as mean ± SD. The unpaired two-tailed *t* test was used for comparisons between two groups. The two-way ANOVA with multiple comparisons between groups was performed to compare multiple groups. GraphPad Prism 7.0 (GraphPad, San Diego, CA, U.S.A.) was used to perform all analyses. The significance threshold was set to *P* values < 0.05.

## Results

### Naringin prevents ox-LDL-induced endothelial injury

Initially, we tested the possible cytotoxic effects of naringin on HUVECs, and observed that at 10, 50, and 100 µM, no significant cell death was induced after 24 h of incubation, while the highest concentration; 200 µM, significantly decreased cell viability by ∼23% (Figure 1A). In addition, 20, 40, 60, and 80 µg/l ox-LDL incubation for 24 h led to a significant dose-dependent decrease in cell viability (Figure 1B), with only 47.5 ± 6.2% cell viability after incubation with 80 µg/l ox-LDL. Pretreatment with 10 µM naringin for 2 h had no significant influence on cell viability. However, that with 50 and 100 µM naringin significantly enhanced ox-LDL-induced HUVEC viability to 58 ± 7.3% and 79 ± 6.5%, respectively (Figure 1C,D). We also examined the effect of naringin on LDH release. Except for the 10 µM concentration, naringin pretreatment (50 and 100 µM) significantly attenuated LDH release in HUVECs (Figure 1E). Thus, 50 and 100 µM naringin were chosen as the experimental concentrations for studying its protective role against HUVEC injury. Our data suggests that naringin plays a protective role against ox-LDL-induced endothelial injury.

RETRACTED

**Figure 1:** Effects of naringin on ox-LDL-induced HUVECs injury Naringin plays a protective role against ox-LDL-induced endothelial injury. Assessment of the dose–response effect of naringin (**A**) and ox-LDL (**B**) on cell viability, using the CCK-8 assay. (**C** and** D**) Representative results and assessment of the dose–response effect of naringin on cell viability in the presence or absence of ox-LDL (80 μg/ml). HUVECs were pretreated with various concentrations of naringin for 2 h, followed by incubation with ox-LDL (80 μg/ml) for 24 h; scale bars: 50 and 10 μm. (**E**) Assessment of the dose–response effect of naringin on LDH release in the presence or absence of ox-LDL (80 μg/ml). Data are presented as mean ± SD, *n* = 6, *P < 0.05, **P < 0.01, and ***P < 0.001 vs. the vehicle-treated control; ^###^*P* < 0.001 vs. the ox-LDL-induced cells.

### Naringin prevents ox-LDL-induced endothelial apoptosis

We further investigated the inhibitory role of naringin in ox-LDL-induced cell apoptosis. The TUNEL assay confirmed the protective effect of naringin against the ox-LDL challenge (Figure 2A). The percentage of TUNEL-positive cells dramatically increased after 80 µg/l ox-LDL. However, a significant dose-dependent decrease was observed in naringin-pretreated cells (Figure 2B). Moreover, flow cytometry results also revealed that the 80 µg/l ox-LDL-induced HUVEC apoptosis was dramatically dose-dependently reversed in naringin-pretreated cells (Figure 2C,D). In essence, naringin inhibits ox-LDL stimulated endothelial apoptosis.

**Figure 2:** Naringin attenuates ox-LDL-induced apoptosis in HUVECs Naringin could inhibits ox-LDL stimulated endothelial apoptosis. HUVECs were pretreated with (50 or 100 µM) naringin for 2 h, followed by treatment with 80 µg/l ox-LDL for 24 h. (**A**) Representative image of TUNEL assay. (**B**) The percentage of TUNEL-positive cells was quantified. (**C**) Apoptosis of HUVECs in different groups was examined with a FITC Annexin V apoptosis kit, via flow cytometry. (**D**) Quantitative data show that ox-LDL increased the apoptotic rate in HUVECs, which was significantly dose-dependently reversed by naringin. Data are presented as mean±SD, *n* = 6, ^###^*P* < 0.001 vs. the control group, **P < 0.01 and ***P < 0.001 vs. the ox-LDL group.

### Naringin inhibits EndMT and the inflammatory response in ox-LDL-induced HUVECs

Immunofluorescent staining showed that incubating HUVECs with ox-LDL decreased the expression of the endothelial marker VE-cadherin, an effect mitigated by naringin (Figure 3A). Western blotting consistently showed that naringin elevated VE-cadherin HUVEC levels, initially down-regulated in the presence of ox-LDL (Figure 3C). The ox-LDL-induced change in HUVEC morphology from cobblestone-like shapes to spindle shapes was significantly reversed in naringin-pretreated cells (Figure 3B). Moreover, Western blotting showed that F-actin protein expression, which was significantly enhanced in ox-LDL-induced HUVECs, was dose-dependently reversed in naringin-pretreated cells (Figure 3D,E). These results suggest that naringin plays an important inhibition role in ox-LDL-induced HUVEC EndMT.

RETRACTED

**Figure 3:** Naringin inhibits the inflammatory response and EndMT in ox-LDL-induced HUVEC cells Naringin inhibits the endothelial damage and the inflammatory response in ox-LDL-induced HUVECs. After pretreated with different concentrations of naringin (50 or 100 µM) for 2 h, cells were exposed to ox-LDL (80 μg/ml) and incubated for 24 h. Immunostaining showed VE-cadherin (**A**) and F-actin (**B**) expression in the HUVECs; scale bar is 10 μm. Green indicates cells labeled with VE-cadherin and F-actin; blue, DAPI. (**C**) Expression of VE-cadherin and F-actin in HUVECs, determined by Western blotting. GAPDH was used as internal control. Representative Western blot bands are shown in panels (**C** and **D**). Quantified VE-cadherin protein expression. (**E**) Quantified F-actin protein expression. (**F**–**H**) qRT-PCR was performed to determine the production of the proinflammatory cytokines IL-1β (F), IL-6 (G), and IL-18 (H) in ox-LDL-induced HUVECs. Data are presented as mean ± SD, *n* = 6, ^###^*P* < 0.001 vs. the control group, *P < 0.01, **P < 0.01, and ***P < 0.001 vs. the ox-LDL group.

To determine if naringin regulates the inflammatory response in ox-LDL-induced HUVECs, we performed qRT-PCR to measure their IL-1β, IL-6, and IL-18 mRNA levels. ox-LDL at 80 µg/l, dramatically enhanced IL-1β, IL-6, and IL-18 mRNA levels in HUVECs, which was significantly dose-dependently attenuated in naringin-pretreated cells (Figure 3F–H).

### Naringin reverses ox-LDL-induced YAP attenuation in HUVECs

RT-PCR results showed that ox-LDL stimulation resulted in dose-dependent attenuated YAP mRNA levels in HUVECs (Figure 4A). Western blotting also showed that ox-LDL stimulation resulted in dose-dependent attenuated YAP protein levels in HUVECs (Figure 4B). Immunofluorescent staining showed that incubating HUVECs with ox-LDL, dose-dependently decreased YAP expression (Figure 4C,D), while Western blotting showed a dose-dependent decrease in ox-LDL-induced YAP protein down-regulation, in naringin-pretreated cells (Figure 4E).

**Figure 4:** Naringin reverses ox-LDL-induced YAP attenuation in HUVECs Naringin reverses dose-dependent decrease in ox-LDL-induced YAP down-regulation, in naringin-pretreated cells. (**A**) qRT-PCR showing that YAP mRNA levels were significantly concentration-dependently reduced by ox-LDL. (**B**) Western blotting was performed to determine YAP protein levels. (**C**) Fluorescence microscopy after immunofluorescent staining with a YAP antibody, followed by FITC-labeled secondary antibody (green, original magnification × 100). The nucleus was stained with DAPI (blue). (**D**) Quantification of the fluorescence intensity of YAP. Data are presented as mean ± SD, *n* = 6, *P < 0.05, **P < 0.01, and ***P < 0.001 vs. the control group. (**E**) After pretreatment with naringin (10, 50 and 100 μM), cells were exposed to ox-LDL (80 μg/ml). Western blotting was performed to determine YAP protein levels. Data are presented as mean±SD, *n* = 6, ^###^*P* < 0.001 vs. the control group, ***P < 0.001 vs. the ox-LDL group.

RETRACTED

### YAP inhibition attenuates the protective effects of naringin against ox-LDL–mediated HUVEC injury

To further investigate the role of YAP on naringin protective effects against ox-LDL–mediated HUVEC injury, we used YAP shRNA to inhibit YAP expression. HUVECs were transfected with YAP shRNA or control shRNA for 48 h, pretreated with naringin (100 µM) for 2 h, and then incubated with ox-LDL (80 µg/l) for 24 h. The results showed that YAP shRNA successfully abolished naringin-induced YAP protein up-regulation in ox-LDL-mediated HUVECs (Figure 5A and B). Moreover, transfection with YAP shRNA reversed the effects of naringin: increased cell viability (Figure 5C), down-regulated LDH release (Figure 5D), and decreased cell apoptosis (Figure 5E,F), compared with the ox-LDL+naringin group. In contrast, transfection with control shRNA had no effect on cell viability, LDH release, and cell apoptosis. These data suggest that the protective role of naringin on ox-LDL–mediated HUVEC injury was at least partially achieved by up-regulating YAP expression.

**Figure 5:** YAP inhibition attenuates naringin protective effects against ox-LDL–mediated HUVEC injury The mechanisms of the protective role of naringin on ox-LDL–mediated HUVEC injury were investigated by down-regulating YAP expression. HUVEC cells were divided into four groups: ox-LDL group, ox-LDL + naringin group, ox-LDL + naringin + shRNA-Con group, and ox-LDL + naringin + shRNA-YAP group. In each group, HUVECs were pretreated with naringin (100 µM) or naringin (100 µM) + shRNA-Con or naringin (100 µM) + shRNA-YAP, for 2 h, then exposed to ox-LDL (80 μg/ml) and incubated for 24 h. (**A** and** B**) Western blotting was performed to determine YAP protein levels. (**C**) Cell viability was determined using the CCK-8 assay. (**D**) LDH activity was quantified. (**E**) TUNEL-positive cells were quantified by TUNEL immunofluorescent staining. (**F**) Apoptotic cells were quantified with a FITC Annexin V apoptosis kit, via flow cytometry. Data are presented as mean ± SD, *n* = 6, ^##^*P* < 0.01 and ^###^*P* < 0.001 vs. the ox-LDL group, **P < 0.01 and ***P < 0.001 vs. the ox-LDL + naringin group.

RETRACTED

## Discussion

It is commonly thought that endothelial cell injury and apoptosis are the basis and initial steps in the pathogenesis of atherosclerosis [19]. Under pathological conditions, chemical stress from harmful substances such as cytokines and oxidized lipids (such as ox-LDL), are known to be key players in endothelial cell injury [8]. ox-LDL-induced endothelial injury is considered a crucial contributor to the pathogenesis and progression of atherosclerosis [20]. Hence, inhibiting ox-LDL-induced endothelial injury may be a novel effective therapeutic approach against atherosclerosis.

In the present study, we evaluated the effect of naringin on ox-LDL-induced HUVEC injury. Previous studies have shown that naringin prevents *in vitro* LDL oxidation via influencing copper binding to LDL [21], probably important in preventing atherosclerosis. Reports have shown the ability of naringin to inhibit monocyte adhesion to endothelial cells induced by TNF-α [22] and high glucose [23]. Naringin also inhibits apoptosis and inflammation in LPS-induced HUVECs [24]. Research by Kim et al. indicated that naringin had no effect on ox-LDL-induced monocyte adhesion [25]. However, whether naringin affects apoptosis, EndMT, and inflammation in ox-LDL-induced HUVECs, and the underlying mechanisms, remain unclear.

Our study revealed that ox-LDL (80 μg/ml) stimulation reduced cell viability and increased LDH release in HUVECs, which was dose-dependently reversed in cells pretreated with naringin for 2 h (50 and 100 μM). Further studies using the CCK-8 assay and flow cytometry indicated that naringin reduced apoptosis. These results suggest that naringin can inhibit ox-LDL-induced cell injury and apoptosis.

It is well known that inflammation, an important biological process, is associated with atherogenesis [26]. Our study demonstrated that naringin inhibited ox-LDL-induced release of inflammatory cytokines such as IL-1β, IL-6, and IL-18, indicating that it attenuated ox-LDL-induced inflammation. These results suggest that naringin can inhibit ox-LDL-induced HUVEC damage by suppressing inflammatory reactions. Previous studies by Bi et al. showed that naringin significantly downregulated the protein or mRNA levels of IL-1, IL-6, and TNF-α, and suppressed LPS-induced inflammation and apoptosis [24], which is consistent with our findings.

RETRACTED

EndMT, characterized by specific endothelial marker loss and mesenchymal marker acquisition, is crucial for atherosclerosis [27]. Western blotting and immunofluorescent staining showed that the endothelial cell marker VE-cadherin was significantly attenuated in ox-LDL-induced HUVECs, a condition that was dramatically reversed by naringin. Moreover, F-actin immunofluorescent staining revealed that ox-LDL induced change in HUVEC morphology, from cobblestone-like shapes to spindle shapes, which was mitigated by naringin treatment. These results indicate that naringin modulated ox-LDL-induced EndMT in HUVECs. Vaccarin, another flavonoid glycoside isolated from vaccariae semen, was initially shown to impede ox-LDL-triggered HUVEC inflammation, EndMT, and apoptosis [28]. Our study suggests that naringin and vaccarin may have similar endothelial protective effects.

Endothelial Cell–Specific Deletion of YAP has been associated with an increase in the expression of inflammatory cytokines like IL-6, TNF-α, and IL-1β [29], which prompted us to investigate the role of YAP in naringin treatment ox-LDL-induced HUVECs. YAP/TAZ are critical in regulating several cellular behaviors, in response to various internal and external stimuli [30]. An increasing number of studies have shown that Hippo–YAP/TAZ signaling has emerged as a new blood vessel development pathway. Azad et al. reported the Hippo–YAP pathway as a critical mediator of vascular endothelial growth factor (VEGF)-induced angiogenesis, and tumor vasculogenic mimicry [31]. Our research found that naringin reversed YAP’s down-regulation caused by ox-LDL, in addition, when shRNA was used to inhibit YAP expression, the cytoprotective and anti-apoptotic naringin function on ox-LDL-induced HUVECs, was inhibited. YAP negatively regulated inflammatory signaling [29] and knockdown of YAP reversed cytoprotective of naringin on ox-LDL-induced HUVECs, which suggest that YAP is a positive modulator in atherosclerosis; however, YAP knockdown attenuated the disturbed flow induction of endothelial cells proliferation and inflammation [32], which indicate that YAP is a negative regulator in atherosclerosis. A possible explanation is that different stimuli activate YAP through different mechanisms, thus play different roles in atherosclerosis. Overall, we confirmed that naringin modulated ox-LDL-induced apoptosis, EndMT, and inflammation *in vitro*, via the YAP pathway.

However, the present study had some limitations, given that no *in vivo* assay was performed to confirm the *in vitro* results. Hence, further *in vivo* experiments should be performed to demonstrate these naringin endothelial effects. In conclusion, the present study determined for the first time that naringin attenuates ox-LDL-induced HUVEC injury by suppressing cell apoptosis, EndMT, and inflammation, via inhibition of the YAP pathway.

RETRACTED

## Abbreviations

EndMT: endothelial–mesenchymal transition
HUVEC: human umbilical vein endothelial cell
ox-LDL: oxidized low-density lipoprotein
YAP: yes-associated protein 1

## References

[1] GuoX., GaoM., WangY., LinX., YangL., CongN.et al. (2018) LDL receptor gene-ablated hamsters: a rodent model of familial hypercholesterolemia with dominant inheritance and diet-induced coronary atherosclerosis. EBioMedicine 27, 214–224 10.1016/j.ebiom.2017.12.01329289533PMC5828369

[2] GimbroneM.A.Jr and García-CardeñaG. (2016) Endothelial cell dysfunction and the pathobiology of atherosclerosis. Circ. Res. 118, 620–636 10.1161/CIRCRESAHA.115.30630126892962PMC4762052

[3] Rafieian-KopaeiM., SetorkiM., DoudiM., BaradaranA. and NasriH. (2014) Atherosclerosis: process, indicators, risk factors and new hopes. Int. J. Prev. Med. 5, 92725489440PMC4258672

[4] KovacicJ.C., DimmelerS., HarveyR.P., FinkelT., AikawaE., KrenningG.et al. (2019) Endothelial to mesenchymal transition in cardiovascular disease: JACC state-of-the-art review. J. Am. Coll. Cardiol. 73, 190–209 10.1016/j.jacc.2018.09.08930654892PMC6865825

[5] LiA., PengW., XiaX., LiR., WangY. and WeiD. (2017) Endothelial-to-mesenchymal transition: a potential mechanism for atherosclerosis plaque progression and destabilization. DNA Cell Biol. 36, 883–891 10.1089/dna.2017.377928920704

[6] KasikaraC., DoranA.C., CaiB. and TabasI. (2018) The role of non-resolving inflammation in atherosclerosis. J. Clin. Invest. 128, 2713–2723 10.1172/JCI9795030108191PMC6025992

[7] YurdagulA.Jr, DoranA.C., CaiB., FredmanG. and TabasI.A. (2018) Mechanisms and consequences of defective efferocytosis in atherosclerosis. Front. Cardiovasc. Med. 4, 86 10.3389/fcvm.2017.0008629379788PMC5770804

[8] LintonM.F., YanceyP.G., DaviesS.S., JeromeW.G., LintonE.F., SongW.L.et al. (2019) The role of lipids and lipoproteins in atherosclerosis. Endotext [Internet]: MDText. com, Inc.https://www.ncbi.nlm.nih.gov/books/NBK343489/

[9] LinF., PeiL., ZhangQ., HanW., JiangS., LinY.et al. (2018) Ox‐LDL induces endothelial cell apoptosis and macrophage migration by regulating caveolin‐1 phosphorylation. J. Cell. Physiol. 233, 6683–6692 10.1002/jcp.2646829323707

[10] BacanlıM., BaşaranA.A. and BaşaranN. (2018) The major flavonoid of grapefruit: naringin, in polyphenols: prevention and treatment of human disease. In Polyphenols: Prevention And Treatment Of Human Disease, 2nd edn(WatsonR., Victor PreedyV. and ZibadiS., eds), pp. 37–44Elsevier: Academic press, Oxford, England

RETRACTED

[11] BurkeA.C., SutherlandB.G., TelfordD.E., MorrowM.R., SawyezC.G., EdwardsJ.Y.et al. (2019) Naringenin enhances the regression of atherosclerosis induced by a chow diet in Ldlr−/− mice. Atherosclerosis 286, 60–70 10.1016/j.atherosclerosis.2019.05.00931102954

[12] RazaviB.M. and HosseinzadehH. (2019) A review of the effects of citrus paradisi (grapefruit) and its flavonoids, naringin, and naringenin in metabolic syndrome, in bioactive food as dietary interventions for diabetes. Phytother. Res.515–543 10.1002/ptr.6573

[13] SalehiB., FokouP.V.T., Sharifi-RadM., ZuccaP., PezzaniR., MartinsN.et al. (2019) The therapeutic potential of naringenin: a review of clinical trials. Pharmaceuticals 12, 11 10.3390/ph12010011PMC646916330634637

[14] Hernández-AquinoE. and MurielP. (2018) Beneficial effects of naringenin in liver diseases: Molecular mechanisms. World J. Gastroenterol. 24, 1679 10.3748/wjg.v24.i16.167929713125PMC5922990

[15] HeJ., BaoQ., YanM., LiangJ., ZhuY., WangC.et al. (2018) The role of Hippo/yes‐associated protein signalling in vascular remodelling associated with cardiovascular disease. Br. J. Pharmacol. 175, 1354–1361 10.1111/bph.1380628369744PMC5866970

[16] AvruchJ., ZhouD., FitamantJ., BardeesyN., MouF. and BarrufetL.R. (2012) Protein kinases of the Hippo pathway: regulation and substrates. In Seminars In Cell And Developmental Biology, Elsevier10.1016/j.semcdb.2012.07.002PMC348901222898666

[17] LvY., KimK., ShengY., ChoJ., QianZ., ZhaoY.-Y.et al. (2018) YAP controls endothelial activation and vascular inflammation through TRAF6. Circ. Res. 123, 43–56 10.1161/CIRCRESAHA.118.31314329794022PMC6014930

[18] LiuT.T., ZengY., TangK., ChenX., ZhangW. and Le XuX. (2017) Dihydromyricetin ameliorates atherosclerosis in LDL receptor deficient mice. Atherosclerosis 262, 39–50 10.1016/j.atherosclerosis.2017.05.00328500865

[19] WuM.-Y., LiC.-J., HouM.-F. and ChuP.-Y. (2017) New insights into the role of inflammation in the pathogenesis of atherosclerosis. Int. J. Mol. Sci. 18, 2034 10.3390/ijms18102034PMC566671628937652

[20] LeivaE., WehingerS., GuzmánL. and OrregoR. (2015) Role of oxidized LDL in atherosclerosis, in Hypercholesterolemia. IntechOpen

[21] NaderiG.A., AsgaryS., Sarraf-ZadeganG.N., GholamN. and ShirvanyH. (2003) Anti-oxidant effect of flavonoids on the susceptibility of LDL oxidation [M]. Vascular Biochem. Springer193–196 10.1007/978-1-4615-0298-2_2712841362

[22] LiW., WangC., PengJ., LiangJ., JinY., LiuQ.et al. (2014) Naringin inhibits TNF-α induced oxidative stress and inflammatory response in HUVECs via Nox4/NF-κ B and PI3K/Akt pathways. Curr. Pharm. Biotechnol. 15, 1173–1182 10.2174/138920101566614111111444225391245

RETRACTED

[23] XiongY., WangG., ZhangJ., WuS., XuW., ZhangJ.et al. (2010) Naringin inhibits monocyte adhesion to high glucose-induced human umbilical vein endothelial cells. Nan fang yi ke da xue xue bao 30, 321–325 20159712

[24] BiC., JiangY., FuT., HaoY., ZhuX. and LuY. (2016) Naringin inhibits lipopolysaccharide-induced damage in human umbilical vein endothelial cells via attenuation of inflammation, apoptosis and MAPK pathways. Cytotechnology 68, 1473–1487 10.1007/s10616-015-9908-327006302PMC4960195

[25] KimS.W., KimC.E. and KimM.H. (2011) Flavonoids inhibit high glucose-induced up-regulation of ICAM-1 via the p38 MAPK pathway in human vein endothelial cells. Biochem. Biophys. Res. Commun. 415, 602–607 10.1016/j.bbrc.2011.10.11522074828

[26] GeovaniniG.R. and LibbyP. (2018) Atherosclerosis and inflammation: overview and updates. Clin. Sci. 132, 1243–1252 10.1042/CS2018030629930142

[27] EvrardS.M., LecceL., MichelisK.C., Nomura-KitabayashiA., PandeyG., PurushothamanK.-R.et al. (2016) Endothelial to mesenchymal transition is common in atherosclerotic lesions and is associated with plaque instability. Nat. Commun. 7, 11853 10.1038/ncomms1185327340017PMC4931033

[28] GongL., LeiY., LiuY., TanF., LiS., WangX.et al. (2019) Vaccarin prevents ox-LDL-induced HUVEC EndMT, inflammation and apoptosis by suppressing ROS/p38 MAPK signaling. Am. J. Transl. Res. 11, 214031105824PMC6511755

[29] LvY., KimK., ShengY., ChoJ., QainZ., ZhaoY.-Y.et al., YAP Controls Endothelial Activation and Vascular Inflammation Through TRAF6. Circul Res. Circresaha 118, 31314310.1161/CIRCRESAHA.118.313143PMC601493029794022

[30] VarelasX. (2014) The Hippo pathway effectors TAZ and YAP in development, homeostasis and disease. Development 141, 1614–1626 10.1242/dev.10237624715453

[31] AzadT., van RensburgH.J., LightbodyE., NeveuB., ChampagneA., GhaffariA.et al. (2018) A LATS biosensor screen identifies VEGFR as a regulator of the Hippo pathway in angiogenesis. Nat. Commun. 9, 1061 10.1038/s41467-018-03278-w29535383PMC5849716

[32] WangK., YehY., NguyenP., LimquecoE., LopezJ., ThorossianS.et al. (2016) Flow-dependent YAP/TAZ activities regulate endothelial phenotypes and atherosclerosis. Proc. Natl Acad. Sci. 113, 11525–11530 10.1073/pnas.161312111327671657PMC5068257

